The article "Influences of Ultrasonic Image-Guided Erector Spinae Plane Block on Postoperative Pulmonary Air Content of Lung Carcinoma Patients Undergoing Thoracoscopic Surgery" was published in 2022. Journal: Comput Math Methods Med.

# Influences of Ultrasonic Image-Guided Erector Spinae Plane Block on Postoperative Pulmonary Air Content of Lung Carcinoma Patients Undergoing Thoracoscopic Surgery

**DOI:** 10.1155/2022/1301361

**Published:** 2022-09-06

**Authors:** Xiuqing Xu, Shengrong Yang, Pei Gao

**Affiliations:** Department of Anesthesiology, Binhai County People's Hospital, Affiliated Hospital of Kangda College of Nanjing Medical University, Yancheng, 224500 Jiangsu, China

## Abstract

To investigate the influences of ultrasonic image-guided erector spinae plane block (ESPB) on postoperative pulmonary air content of lung carcinoma patients undergoing thoracoscopic surgery, 42 patients performed with thoracoscopic radical surgery for lung carcinoma were selected. The patients in the experimental group were performed with ultrasound-guided unilateral ESPB and intravenous general anesthesia. The patients in the control group only underwent intravenous anesthesia. The changes in postoperative pulmonary air content between the two groups were compared. After that, all included patients were divided into the experimental (senior) group (13 cases), the experimental (adult) group (8 cases), the control (senior) group (11 cases), and the control (adult) group (10 cases) according to age. The changes in postoperative pulmonary air content of patients in the four groups were compared. The results showed that lung ultrasound score (LUS) of patients in experimental group was 6.4 ± 3.2 points 0.5 hour after catheter extraction and LUS was 4.1 ± 2.3 points 20 to 30 hours. Both scores were remarkably lower than those of patients in control group (*P* < 0.05). LUS of lower left anterior area, upper left posterior area, lower left posterior area, upper right posterior area, and lower right posterior area of patients in experimental group was all apparently lower than those in control group 0.5 hour after catheter extraction (*P* < 0.05). LUS of upper left posterior area, lower left posterior area, lower right anterior area, upper right posterior area, and lower right posterior area of patients in experimental group was all remarkably lower than those in control group 20 to 30 hours after surgery (*P* < 0.05). LUS of senile patients and middle-aged patients in experimental group 0.5 hour after catheter extraction was 8.01 ± 2.48 points and 5.93 ± 3.91 points, respectively, which were both notably lower than those in control group (*P* < 0.05). Ultrasound-guided ESPB exerted fewer influences on lung and could effectively improve postoperative pulmonary air content among patients. Hence, it was worthy of clinical promotion.

## 1. Introduction

Lung carcinoma is one of the commonest malignant tumors. Over the past 50 years, the incidence of lung carcinoma has been rising year by year [1]. The cause of lung carcinoma is still not very clear. As population aging and environmental pollution gradually become serious, the incidence and mortality of lung carcinoma will further increase. At present, the main clinical treatment method for lung carcinoma is surgical tumor resection. In the early stage of lung carcinoma, therapeutic goal can be achieved by surgical treatment [2]. Thoracoscopic surgery is characterized by small incision, less trauma, and good effect. It is replacing most traditional thoracotomy incisions [3]. Thoracic surgery results in acute postoperative pain, which is related to muscle separation at incision, rib shrinkage, rib resection, and damage to the intercostal nerve. Poor pain management may aggravate postoperative pulmonary dysfunction among patients [4]. During thoracoscopic surgery, the stress reaction caused by surgical trauma is reduced. However, patients tend to weaken the range of respiratory movement and reduce coughing, expectoration, and turning over if postoperative analgesia is poor. As a result, the risk of postoperative atelectasis and lung infection is increased [5].

The article "Influences of Ultrasonic Image-Guided Erector Spinae Plane Block on Postoperative Pulmonary Air Content of Lung Carcinoma Patients Undergoing Thoracoscopic Surgery" was published in 2022. Journal: Comput Math Methods Med.

After thoracic surgery, it is difficult to achieve the best analgesic effect by adopting a single analgesic program. The increase of the dose of opioids results in the growth of the incidence of nausea, vomiting, and other adverse reactions [6]. Local anesthetic shows good analgesic effect and high safety. The application of multimode analgesic methods can help patients recover as soon as possible after surgery [7]. Thoracic epidural block and thoracic paraspinal nerve block are the gold standards of regional analgesia during thoracotomy. According to relevant studies, pain score is affected to some extent [8]. In recent years, the development of ultrasound visualization technology promotes the popularization of nerve block anesthesia. With the guidance of ultrasound, nerve block takes effect in shorter time. Besides, nerve block operation is less time-consuming, success rate is increased, and the incidence of related complications is reduced [9]. Erector spinae plane block (ESPB) is explained as follows. According to different types of surgeries, the corresponding spinal nerve segment is selected, and local anesthetic is injected into fascia in erector spinae to block the nerve in the fascia using appropriate methods. As a result, analgesic effects are shown [10]. Some studies demonstrate that ultrasound-guided ESPB has the similar analgesic effect with paravertebral block. In contrast, it is easier to perform ultrasound-guided ESPB with less time [11].

The article "Influences of Ultrasonic Image-Guided Erector Spinae Plane Block on Postoperative Pulmonary Air Content of Lung Carcinoma Patients Undergoing Thoracoscopic Surgery" was published in 2022. Journal: Comput Math Methods Med.

Some studies show that different levels of postoperative damages to gas exchange or respiratory mechanics occur among all patients even if their pulmonary function is normal without other diseases before anesthesia surgery. The incidence of atelectasis is about 90% [12]. The main cause is that muscular relaxants used for general anesthesia, especially long-acting muscular relaxants, inhibit the function of patients' respiratory muscle, which leads to the reduction in lung air flow in patients' bodies. To deepen anesthesia, heavy use of anesthetic inhibits the excitatory response of the ventilator. In addition, the use of general anesthetic leads to the increased permeability of pulmonary capillary as well as the decreased content of macrophage in patients' bodies and inhibits the release of active substances on the surface of pulmonary alveoli [13]. In addition, adjuvant mechanical ventilation is required because anesthesia inhibits patients' respiratory function. However, respiratory system resistance is increased without muscle tone in this case. During mechanical ventilation, pulmonary alveoli collapses, shearing injury occurs, and pulmonary compliance changes abnormally. A variety of reasons lead to the reduction in patients' functional residual capacity and lung air content. What is worse, these reasons cause pulmonary vascular shunt and pulmonary gas exchange cannot occur, which further develops into atelectasis [14].

Therefore, the patients undergoing thoracoscopic radical surgery for lung carcinoma were selected and performed with ultrasound-guided ESPB anesthesia method as well as intravenous anesthesia method. The changes in postoperative lung air content of patients were compared, and the influences of ultrasound-guided ESPB anesthesia on postoperative lung air content of patients undergoing thoracoscopic radical surgery for lung carcinoma were investigated to provide reference values for subsequent clinical surgical treatment of lung carcinoma and improve therapeutic effect.

## 2. Research Methods

### 2.1. Objects

Forty-two patients undergoing thoracoscopic radical surgery for lung carcinoma (55 ± 4.3 years old) in hospital were selected. Their body mass index (BMI) was 22 ± 1.5 kg/m^2^. They were randomly divided into two groups. 21 patients in control group were performed only with intravenous general anesthesia. 21 patients in experimental group underwent ultrasound-guided unilateral ESPB and intravenous general anesthesia. Further grouping: according to whether the patient was 65 years old or above, they were divided into elderly group and middle-aged group, including experimental (elderly) group (13 cases), experimental (adult) group (8 cases), control (elderly) group (11 cases), and control (adult) group (10 cases). All included research objects had signed informed consent forms, and this study had been approved by ethics committee of hospital.

The article "Influences of Ultrasonic Image-Guided Erector Spinae Plane Block on Postoperative Pulmonary Air Content of Lung Carcinoma Patients Undergoing Thoracoscopic Surgery" was published in 2022. Journal: Comput Math Methods Med.

Inclusion criteria: patients with American Society of Anesthesiologists (ASA) level I and II and BMI below 30 kg/m^2^; patients with generally normal pulmonary function on admission; patients without previous history of radiotherapy and chemotherapy and using antipsychotic drug, antisympathetic drug, antipsychotic drug, and drugs interfering with adrenal function for a period of time before surgery; patients who could normally understand and be cooperative throughout the experiment.

Exclusion criteria: patients with hypertension level at II or above and complicated cerebrovascular disease; patients with complicated empyema and puncture site infection; patients with serious circulation system disease; patients with abnormal curvature of the spine and space occupying lesion of erector spinae; patients with serious liver and renal insufficiency.

### 2.2. Anesthesia Method

The detailed survey of patients' condition was carried out, and the risks and possible accidents of surgical anesthesia were explained to patients. Relevant knowledge about anesthesia were introduced to patients, and they were instructed to sign informed consent forms. Routine fasting lasted for 8 hours and abstinence lasted for 4 hours before surgery.

Anesthesia methods were explained as follows. After entering operating room, upper limb venous channel was routinely established. 10 ml/kg sodium lactate Ringer's injection was infused. Besides, mask oxygen inhalation was implemented, and oxygen flow was 2 L/min. Under local anesthesia, radial artery puncture was performed for invasive arterial blood pressure monitoring. Puncture and catheterization were performed for right internal jugular vein for the preparation of intraoperative fluid replenishment and venous blood extraction. Besides, electrocardio, pulse, and oxygen saturation were routinely monitored. Patients in experimental group were instructed to take lateral position and receive single ESPB at T5 horizontal transverse process under the guidance of ultrasound. 25 mL of 0.4% ropivacaine was used for local anesthesia. After 20 minutes, ice method was adopted to test block plane at the anterior axillary line of the affected side and assess if puncture was routine. If the plane was less than three segments, puncture failed and was not included in the research. The patients in control group were performed only with intravenous general anesthesia. Before the anesthesia induction, 100 mL physiological saline was injected with 0.5 *μ*g/kg dexmedetomidine hydrochloride, and intravenous drip was carried out within 15 minutes. After that, all patients received intravenous general anesthesia and the venous injection of 1.5-2.0 mg/kg propofol, 0.5 *μ*g/kg sufentanil, and 1.5 mg/kg cis-atracurium. Double lumen bronchial intubation was implemented, and adjuvant mechanical ventilation was carried out after the accurate positioning of fiber bronchoscope. Intravenous micropump was used to pump propofol (4-6 mg/kg/h) and remifentanil (0.1-1 *μ*g/kg/h) to maintain anesthesia. Cis-atracurium was injected intermittently. According to the stimulation intensity, cyclic change, and bispectral index of intraoperative operation, the dosage of propofol and remifentanil was adjusted, and the value of bispectral index was kept between 40 and 60. Normally, blood pressure should fluctuate within ±20% of basic blood pressure. Insulation measure should be taken during the surgery. Target-oriented transfusion treatment was adopted, and PetCO_2_ was kept between 30 and 40 mmHg. 100 g flurbiprofen axetil was offered for patients to perform analgesic cohesion half an hour before skin suture. After surgery, the patients in the two groups carried out patient-controlled intravenous analgesia (PCIA). Analgesic pump formulation was as follows. 1.0 *μ*g/mL sufentanil, 32 mg ondansetron hydrochloride tablets, and physiological saline were diluted to 100 mL. Background infusion was 2.5 mL/h per time followed by 2.5 mL, and the lock time was 25 minutes. After the surgery, routine vital sign monitoring and extubation were performed according to patients' situation.

The article "Influences of Ultrasonic Image-Guided Erector Spinae Plane Block on Postoperative Pulmonary Air Content of Lung Carcinoma Patients Undergoing Thoracoscopic Surgery" was published in 2022. Journal: Comput Math Methods Med.

Ultrasound-guided ESPB was explained as follows. In the experiment, ultrasound-guided unilateral ESPB based on minor axis in-plane technique was utilized. Based on ultrasonic imaging, the trajectory of the needle tip in the needle track could be accurately seen. The needle tip reached the surface of transverse process and the deep surface of erector spinae safely and conventionally. Patients were asked to take lateral position. T5 spinous process was determined and then labeled. Conventional disinfection and skin preparation were performed. After that, the ultrasonic probe was placed longitudinally parallel to the spine at 2 to 3 cm outside T5 spinous process. Through ultrasonic screen imaging, trapezius muscle, rhomboideus, erector spinae, and T5 transverse process could be accurately observed from top to bottom. A 22G puncture needle was inserted from head to end. The needle tip position was determined by injecting 1-2 mL of physiological saline after no air or blood was pumped back. Next, the local anesthetic solution was injected into the surface of T5 transverse process and the deep surface of erector spinae. If the local anesthetic solution diffused in the plane of erector spinae fascia and erector spinae elevated, block operation was successful. After 20 minutes, ice method was adopted to feel and test the block plane at anterior axillary line level.

The article "Influences of Ultrasonic Image-Guided Erector Spinae Plane Block on Postoperative Pulmonary Air Content of Lung Carcinoma Patients Undergoing Thoracoscopic Surgery" was published in 2022. Journal: Comput Math Methods Med.

### 2.3. Division of Lung Ultrasound Regions

Ultrasound equipment was used. Twelve division method was adopted for examination [15, 16]. Bilateral anterior axillary line and posterior axillary line were set as the boundary. Lung area was divided into anterior, lateral, and posterior areas. Besides, bilateral nipple connection lines were set as the boundary. The anterior, lateral, and posterior areas were divided into upper left anterior area, lower left anterior area, upper left lateral area, lower left lateral area, upper left posterior area, lower left posterior area, upper right anterior area, upper right posterior area, upper right lateral area, lower right lateral area, upper right posterior area, and lower right posterior area. A low-frequency convex array probe with the frequency of 2 to 5 MHz was used to collect ultrasonic images from 12 areas of the whole lung. During the collection, the pulmonary ultrasonic images of each area were preserved for 15 s. The sites where pulmonary air content images changed most obviously were collected firstly. If the collected ultrasonic images were not clear and they could not display the real change of patients' lungs, more videos needed to be recorded or more images should be collected.

### 2.4. Ultrasound Image Scoring

After imaging acquisition, the semiquantitative scoring standard was adopted to pulmonary ultrasonic signs. According to LUS, the severity of the changes in pulmonary air content was determined. The score for each pulmonary ultrasonic area ranged between 0 and 3 points. The total score of all 12 areas in the whole lung ranged between 0 and 36 points. 0 point indicated no abnormality in air content. A lower LUS suggested that the difference in the change of pulmonary air content was less significant and higher level of pulmonary air content. A higher LUS meant more remarkable reduction in pulmonary air content and worse condition, as displayed in Table 1.

### 2.5. Statistical Methods

SPSS 22.0 statistical software was utilized for analysis. Measurement data were expressed with mean ± standard deviation (^−^*x* ± *s*). General data were analyzed with independent sample *t* test. Paired sample *t* test was used to compare pulmonary LUS of healthy volunteers at different time points. *P* < 0.05 indicated that the difference showed statistical meaning.

## 3. Results

### 3.1. General Data

Age, BMI, ASA level, anesthesia time, and other general data of patients in the two groups demonstrated no statistical differences (*P* > 0.05), as displayed in Table 2.

The article "Influences of Ultrasonic Image-Guided Erector Spinae Plane Block on Postoperative Pulmonary Air Content of Lung Carcinoma Patients Undergoing Thoracoscopic Surgery" was published in 2022. Journal: Comput Math Methods Med.

### 3.2. Lung Ultrasound Images

Images were acquired when patients were visited on the morning of surgery day or the day before surgery. In analysis of a 56-year-old male patient, images were acquired 0.5 hour after the tracheal tube was removed and postoperative extubation was indicated. Images were acquired 20 to 30 hours after surgery, indicating that ultrasound can clearly show the lung disease in the lungs (Figure 1).

### 3.3. Whole Lung LUS of Patients

The difference in LUS of patients in the two groups on the morning of surgery day revealed no statistical meaning (*P* > 0.05). LUS of patients in experimental group (6.4 ± 3.2 points) was remarkably lower than that of patients in control group (10.3 ± 3.8 points) 0.5 hour after catheter extraction, and the difference was significantly significant (*P* < 0.05). LUS of patients in experimental group (4.1 ± 2.3 points) was notably lower than that of patients in control group (7.7 ± 2.9 points) 20 to 30 hours after surgery, and the difference showed statistical meaning (*P* < 0.05), as illustrated in Figure 2.

### 3.4. LUS of 12 Pulmonary Areas of Patients in the Two Groups

Figure 3(a) is the upper left anterior region; Figure 3(b) is the LUS score results of the lung region in the lower left region at different times, 20-30 hours after the operation, the LUS score of the lower left anterior area in the control group was higher than that in the experimental group.

Figure 3(c) is the LUS score results of the lung region in the upper left region at different times. The figure shows that the upper left area of the control group is higher than that of the observation group in the three time periods.

Figure 3(d) is the lung region in the lower left region at different times. LUS score results: the figure shows that the upper left area of the control group is higher than that of the observation group in the three time periods.

Figure 3(e) is the LUS score results of the left upper posterior region at different times, the LUS score in the lower left area of the observation group was significantly lower than that of the experimental group at 0.5 hours and 20-30 hours after extubation (*P* < 0.05).

Figure 3(f) is the LUS score results of the left lower posterior region at different times. The LUS score in the lower left area of the observation group was significantly lower than that of the experimental group at 0.5 hours and 20-30 hours after extubation (*P* < 0.05).

Figure 4(a) is the upper right anterior area; Figure 4(b) is the LUS score results of the lower right anterior area at different times. The LUS score of the lower right anterior area of the observation group was higher than that of the control group at 0.5 hours after extubation and 20-30 hours after operation.  Figure 4(c) is the LUS score results of the upper right area at different times. On the day of operation and 20-30 hours after extubation, the LUS score in the upper right area of the control group was higher than that of the observation group, but the LUS score of the upper right area of the control group was lower than that of the observation group at 0.5 hours after extubation.  Figure 4(d) is the lower right area at different times. The LUS score results of the lung area: the lower right area of the control group was higher than that of the experimental group in the three time periods, but the experimental group was significantly lower than the control group at 20-30 hours after surgery (*P* < 0.05).  Figure 4(e) is the upper right posterior area. The LUS score in the upper right posterior area of the observation group was significantly lower than that of the control group at 0.5 h and 20-30 hours after extubation (*P* < 0.05).  Figure 4(f) is the LUS score results of the lung area at different times in the lower right posterior area. The LUS score in the lower right posterior area of the observation group was significantly lower than that of the control group at 0.5 h after extubation and 20-30 hours after operation (*P* < 0.05).

The article "Influences of Ultrasonic Image-Guided Erector Spinae Plane Block on Postoperative Pulmonary Air Content of Lung Carcinoma Patients Undergoing Thoracoscopic Surgery" was published in 2022. Journal: Comput Math Methods Med.

### 3.5. Whole Lung LUS of Patients at Different Age Groups

The differences in LUS of patients in the four groups on the morning of surgery day all showed no statistical meaning (*P* > 0.05). LUS of elderly patients in experimental group (8.01 ± 2.48 points) was obviously lower than that of elderly patients in control group (11.96 ± 3.08 points) 0.5 hour after catheter extraction, and the difference had statistical meaning (*P* < 0.05). LUS of middle-aged patients in experimental group (5.93 ± 3.91 points) was remarkably lower than that of middle-aged patients in control group (9.27 ± 3.06 points), and the difference demonstrated statistical meaning (*P* < 0.05). LUS of elderly patients in experimental group (5.68 ± 3.29 points) was dramatically lower than that of elderly patients in control group (8.22 ± 3.05 points) 20 to 30 hours after surgery, and the difference had statistical meaning (*P* < 0.05). LUS of middle-aged patients in experimental group (3.47 ± 3.16 points) was remarkably lower than that of middle-aged patients in control group (7.05 ± 4.02 points), and the difference revealed statistical meaning (*P* < 0.05), as shown in Figure 5.

The article "Influences of Ultrasonic Image-Guided Erector Spinae Plane Block on Postoperative Pulmonary Air Content of Lung Carcinoma Patients Undergoing Thoracoscopic Surgery" was published in 2022. Journal: Comput Math Methods Med.

### 3.6. LUS of 12 Pulmonary Areas of Patients at Different Age Groups in Experimental Group

Figure 6(a) is the upper left anterior region; Figure 6(b) is the LUS score results of 12 lung regions of patients in different age groups in the lower left region. On the day of surgery and 20-30 hours after surgery, the LUS score of the elderly patients in the experimental group was higher than that of the young patients.  Figure 6(c) is the LUS score results of 12 lung regions of patients of different age groups in the upper left region, the scores of the upper left area of the young patients in the experimental groups in the three time periods were significantly lower than those of the elderly patients (*P* < 0.05).  Figure 6(d) is the LUS score results of 12 lung areas of patients in different age groups in the lower left area, the LUS scores in the lower left area of the young group patients were lower than those of the elderly group on the day of surgery and 20-30 hours after the operation.  Figure 6(e) is the LUS score results of 12 lung areas of patients in different age groups in the upper left posterior area, 0.5 hours after extubation and 20-30 hours after surgery, the score of the left upper posterior area in the youth group was lower than the LUS score in the elderly group.  Figure 6(f) is the LUS score of 12 lung areas of patients in different age groups in the lower left posterior area result. At 0.5 hours after extubation and at 20-30 hours after operation, the scores of the left lower posterior area of the youth group were significantly lower than the LUS scores of the elderly group (*P* < 0.05).

Figure 7(a) is the upper right anterior region. The LUS score of the upper right anterior area of the youth group was higher than that of the elderly group after extubation for half an hour, and the score of the elderly group after extubation for 20-30 hours was higher than that of the youth group; Figure 7(b) is the LUS score results of 12 lung regions of patients in different age groups in the lower right region. The LUS score of the elderly group was higher than that of the young group after half an hour of extubation, and the difference was significant (*P* < 0.05).  Figure 7(c) is the LUS score results of 12 lung regions of patients in different age groups in the upper right region, in the three time periods, the scores of the upper right corner of the elderly group were higher than those of the control group, but after 0.5 hours of extubation, the difference was significant (*P* < 0.05).  Figure 7(d) is the LUS score results of 12 lung areas of patients in different age groups in the lower right area. Half an hour after extubation and 20-30 minutes after the operation, the LUS score in the lower right area of the elderly group was higher than that of the young group; half an hour after extubation and 20-30 minutes after the operation, the LUS score in the lower right area of the elderly group was higher than that of the young group.  Figure 7(e) is the LUS score results of 12 lung areas of patients in different age groups in the upper right posterior area; half an hour after extubation and 20-30 minutes after the operation, the LUS score in the upper right posterior area of the elderly group was higher than that of the young group, and the difference was significant (*P* < 0.05).  Figure 7(f) is the 12 lung areas of patients in different age groups in the lower right posterior area district LUS score results. Half an hour after extubation and 20-30 minutes after the operation, the LUS score in the lower right posterior area of the elderly group was higher than that of the young group, and the difference was significant (*P* < 0.05).

The article "Influences of Ultrasonic Image-Guided Erector Spinae Plane Block on Postoperative Pulmonary Air Content of Lung Carcinoma Patients Undergoing Thoracoscopic Surgery" was published in 2022. Journal: Comput Math Methods Med.

## 4. Discussion

In recent years, ESPB is usually used for the combined anesthesia and multimodal analgesia for abdominal, thoracic, pediatric, and orthopedic surgery [17]. Ultrasound-guided ESPB operation is simple. However, some studies showed that pulmonary air content of most patients changed abnormally, and even atelectasis occurred after general anesthesia surgery with the continuous development and improvement of medical technology and the further study on postoperative lung complications among patients [18]. Hence, ESPB block method was adopted to investigate its influences on postoperative pulmonary air content of patients undergoing thoracoscopic surgery for lung carcinoma, which provided reference values for subsequent clinical surgical treatment for patients with lung carcinoma.

According to the research results, LUS of patients in experimental group 0.5 hour after catheter extraction and 20 to 30 hours after surgery was remarkably lower than those of patients in control group (*P* < 0.05). LUS scoring result 0.5 hour after catheter extraction suggested that the scores for lower left lateral area, upper left posterior area, lower left posterior area, upper right posterior area, and lower right posterior area of patients in experimental group were all notably lower than those of patients in control group (*P* < 0.05). LUS scoring result 20 to 30 hours after surgery indicated that the scores for upper left posterior area, lower left posterior area, lower right lateral area, upper right posterior area, and lower right posterior area of patients in experimental group were significantly lower than those of patients in control group (*P* < 0.05). According to relevant studies, postoperative continuous adjuvant positive airway pressure ventilation could effectively reduce LUS score and prevent atelectasis [19]. Hence, ESPB could effectively improve postoperative lung air content among patients compared with single intravenous general anesthesia.

The article "Influences of Ultrasonic Image-Guided Erector Spinae Plane Block on Postoperative Pulmonary Air Content of Lung Carcinoma Patients Undergoing Thoracoscopic Surgery" was published in 2022. Journal: Comput Math Methods Med.

LUS of elderly patients and middle-aged patients in experimental group 0.5 hour after catheter extraction and 20 to 30 hours after surgery was remarkably lower than those of patients in control group (*P* < 0.05). LUS of upper left lateral area of adult patients in experimental group on the morning of surgery day was notably lower than that of elderly patients in experimental group. The scores for upper left lateral area, lower left posterior area, lower right anterior area, upper right lateral area, upper right posterior area, and lower right posterior area of middle-aged patients in experimental group 0.5 hour after catheter extraction were all significantly lower than those of patients in control group (*P* < 0.05). LUS scoring result 20 to 30 hours after surgery revealed that the scores for upper left lateral area, lower left lateral area, lower left posterior area, upper right posterior area, and lower right posterior area of patients in experimental group was all obviously lower than those of patients in control group (*P* < 0.05). The above research results demonstrated that the reduction in postoperative pulmonary air content among senior patients was more remarkable than that among adult patients with higher incidence. The research results were consistent with the conclusion that the incidence of postoperative pulmonary complications among senior patients was relatively higher drawn by Ledowski et al. [20].

## 5. Conclusion

The experiment results showed that both intravenous general anesthesia and ultrasound-guided erector spinae block anesthesia resulted different levels of reduction in pulmonary air content. Compared with that among adult patients, the incidence of the reduction in postoperative pulmonary air content was higher among senior patients. Besides, ultrasound-guided ESPB had fewer influences on postoperative pulmonary air content and improved postoperative pulmonary air content among patients. Due to the impacts of research conditions, the selected sample size is small and the research lasted for a short time, which resulted in insignificant differences between some results. Hence, further study was needed. To sum up, ultrasound-guided ESPB was conducive to improving postoperative pulmonary air content among patients with application values.

## Figures and Tables

**Figure 1:** Pulmonary ultrasound. (a) Ultrasonic image 0.5 hours after extubation. (b) Ultrasonic image 20 hours after surgery.

The article "Influences of Ultrasonic Image-Guided Erector Spinae Plane Block on Postoperative Pulmonary Air Content of Lung Carcinoma Patients Undergoing Thoracoscopic Surgery" was published in 2022. Journal: Comput Math Methods Med.

**Figure 2:** Comparison of whole lung LUS. I: the day of surgery; II: 0.5 h after extubation; III: 20-30 h after operation. ∗Compared with control group, *P* < 0.05.

**Figure 3:** Comparison of left lung LUS scores. I: the day of surgery; II: 0.5 h after extubation; III: 20-30 h after operation. (a) The upper left anterior region. (b) The LUS score results of the lung region in the lower left region at different times. (c) The LUS score results of the lung region in the upper left region at different times. (d) The lung region in the lower left region at different times. (e) The LUS score results of the left upper posterior region at different times. (f) The LUS score results of the left lower posterior region at different times. ∗Compared with control group, *P* < 0.05.

**Figure 4:** Comparison of right lung LUS scores. I: the day of surgery; II: 0.5 h after extubation; III: 20-30 h after operation. (a) The upper right anterior area. (b) The LUS score results of the lower right anterior area at different times. (c) The LUS score results of the upper right area at different times. (d) The lower right area at different times. (e) The upper right posterior area. (f) The LUS score results of the lung area at different times in the lower right posterior area. ∗Compared with control group, *P* < 0.05.

**Figure 5:** Whole lung LUS of patients at different age groups. I: the day of surgery; II: 0.5 h after extubation; III: 20-30 h after operation. ∗Compared with control group, *P* < 0.05.

**Figure 6:** Comparison of left lung LUS scores of patients at different age groups. I: the day of surgery; II: 0.5 h after extubation; III: 20-30 h after operation. (a) The upper left anterior region. (b) The LUS score results of 12 lung regions of patients in different age groups in the lower left region. (c) The LUS score results of 12 lung regions of patients of different age groups in the upper left region. (d) The LUS score results of 12 lung areas of patients in different age groups in the lower left area. (e) The LUS score results of 12 lung areas of patients in different age groups in the upper left posterior area. (f) The LUS score of 12 lung areas of patients in different age groups in the lower left posterior area. ∗Compared with elderly group, *P* < 0.05.

**Figure 7:** Comparison of right lung LUS of patients at different age groups. I: the day of surgery; II: 0.5 h after extubation; III: 20-30 h after operation. (a) The upper right anterior region. (b) The LUS score results of 12 lung regions of patients in different age groups in the lower right region. (c) The LUS score results of 12 lung regions of patients in different age groups in the upper right region. (d) The LUS score results of 12 lung areas of patients in different age groups in the lower right area. (e) The LUS score results of 12 lung areas of patients in different age groups in the upper right posterior area. (f) The 12 lung areas of patients in different age groups in the lower right posterior area district LUS score. ∗Compared with elderly group, *P* < 0.05.

The article "Influences of Ultrasonic Image-Guided Erector Spinae Plane Block on Postoperative Pulmonary Air Content of Lung Carcinoma Patients Undergoing Thoracoscopic Surgery" was published in 2022. Journal: Comput Math Methods Med.

**Table 1:** Scoring standard for pulmonary ultrasonic images.

Image presentation	Scores (value)
Clear A line and lung sliding or 0 to 2 B lines	0
3 or more B lines or small subpleural consolidation separated by smooth pleura line	1
Multiple complicated B lines or they were thickened, and small subpleural consolidation separated by irregular pleura line	2
Solid lung disease	3

**Table 2:** General data on patients.

Groups	Experimental group (21 patients)	Control group (21 patients)
Age (years old)	54 ± 5.8	56 ± 6.2
Gender (male/female)	10/11	8/13
BMI (kg/m^2^)	21 ± 3.6	22 ± 2.4
ASA level (case, I/II)	6/15	9/12
Anesthesia time (min)	128.3 ± 36.7	125.8 ± 38.2

## Data Availability

The data used to support the findings of this study are available from the corresponding author upon request.
